The article "Clinicopathologic features of triple negative breast cancers: an experience from Pakistan" was published in 2014. Journal: Diagn Pathol.

# Clinicopathologic features of triple negative breast cancers: an experience from Pakistan

**DOI:** 10.1186/1746-1596-9-43

**Published:** 2014-02-28

**Authors:** Atif Ali Hashmi, Muhammad Muzzammil Edhi, Hanna Naqvi, Naveen Faridi, Amna Khurshid, Mehmood Khan

**Affiliations:** 1 Department of Histopathology, Liaquat National Hospital and Medical College, Karachi, Pakistan; 2 Liaquat National Hospital and Medical College, Karachi, Pakistan; 3 Dhaka Medical College, Dhaka, Bangladesh

**Keywords:** Triple negative breast cancer, Basal breast cancer, ER, PR, Her2neu

## Abstract

**Background:**

Young age breast cancers are quite prevalent in our setup, a significant number of which exhibit triple negative phenotype. These cancers behave in an aggressive fashion and unresponsive to targeted adjuvant therapy. We aimed to evaluate clinical and histopathologic features of triple negative cancers in our population.

**Methods:**

We retrospectively evaluated 1104 cases of primary breast cancers. Immunohistochemical studies for ER, PR and Her2neu followed by Her2neu gene amplification by FISH testing were done to identify 205 (18.6%) cases of triple negative breast cancers.

**Results:**

Mean age for triple negative breast cancer patients was 48.4 years (±12.3) and 60% of patients were diagnosed at less than 50 years of age. Although ductal carcinoma was the most frequent histologic type, a meaningful number of cases exhibited metaplastic and medullary like features (10.7% and 5.9% respectively). Similarly geographic necrosis involving more than 40% of tumor and extensive lymphocytic infiltration was a considerable finding. Mean Ki67 index was 45.2% (±25.2) and as a reflection of tumor grade, a significantly higher proportion of cases (66.3%) were under high risk Ki67 category (>30%).

**Conclusion:**

Triple negative breast cancers typify high grade breast cancers with a higher frequency of atypical medullary and metaplastic histologies. Their prevailing occurrence at a younger age raises question of under lying BRCA mutations in our population. Therefore, we suggest that risk factors including BRCA 1 mutations should be uncovered in reproductive age group breast cancers especially those disclosing basal like phenotype.

**Virtual slides:**

The virtual slide(s) for this article can be found here: http://www.diagnosticpathology.diagnomx.eu/vs/9042440621102239.

## Introduction

Gene expression profiling studies put a new insight into breast cancer classification beyond traditional histologic sub-typing and grading. These newly defined luminal, Her2neu and basal molecular subtypes of breast cancer in addition to being a powerful indicator of prognosis are also predictive of adjuvant hormonal and chemotherapeutic response [1,2]. Among these, basal type breast cancers are associated with worst prognostic and clinical profile especially if not detected at an early age. They comprise 15-20% of breast cancers and show low expression of ER, PR and Her2neu genes. Basal cancers derived its name by its origin from basal epithelial cells of breast tissue and are thus typified by high expression of basal epithelial cytokeratins [3]. Basal cancers are affiliated with an abnormal DNA damage response pathway with an ancillary elevated proliferation gene expression. Although basal cancer subtype was originally defined by gene expression profiling, however it was suggested that an analogous ascertainment can be made by immunohistochemical (IHC) techniques [4]. According to that annotation, triple negativity for ER, PR and Her2neu elucidate basal type breast cancers with high expression of basal cytokeratins [5]. Majority of triple negative breast cancers by IHC were found to be of basal like phenotype by gene expression profiling, however Fluorescent Insitu hybridization (FISH) testing is recommended by College of American Pathologists (CAP) for intermediate IHC expression of Her2neu [6].

Breast cancer is most frequent cancer of women in Karachi, accounting for one-third of the cancers in the females. The incidence of breast cancer is extremely high in Karachi and second highest in Asia after Israel [7]. A total of 698 cases of breast cancer were registered from Karachi south over a duration of 3 years from 1995-1997 with a crude incidence rate of 33.1%. The incidence of reproductive age breast cancer in karachi is the highest reported globally [8].

Basal cancers have a unique demographic and racial profile, with high rate of occurrence contemplated in Asian and African American women [9]. A comparative study conducted in United States revealed a higher frequency of hormone receptor negative breast cancers in Asian women compared to Caucasians [10]. Analogously a higher frequency of basal cancers was also demonstrated in Chinese women [11]. While the exact incidence of basal cancers in Pakistani population is not characterized, it is well established that frequency of reproductive age breast cancer is considerably higher than the western population [12,13]. As a reason for this happening is not known and pathologic parameters of younger age breast cancer is not well elucidated in our setup, therefore we aimed to determine the frequency and clinicopathologic parameters of triple negative breast cancers in our population which usually show a targeted racial and age preference.

## Methods

We retrospectively analyzed 1104 cases of primary breast cancers treated at Liaquat National Hospital from January 2010 till December 2012 over duration of 3 years. Approval from institutional research and ethical review committee was taken antecedent to conducting the study. Patients after provisional diagnosis of breast cancer underwent trucut biopsies, modified radical mastectomy and breast conservative surgeries. All non–epithelial tumors were excluded from the study. Histologic type of tumors was determined by WHO classification of breast tumors and graded by Modified Bloom-Richardson grading system. Immunohistochemical testing for ER, PR, Her2neu and Ki67 was applied on all cases. A total of 158 out of 1104 cases were negative with ER and PR antibodies and either negative or weak (1+) positive with Her2neu antibody. Total 68 cases were intermediate (2+) positive for Her2neu with negative ER and PR. Therefore subsequent FISH testing was performed on these 68 cases, out of which 19 cases showed Her2neu gene amplification, 2 cases were equivocal and 47 cases were negative for Her2neu gene amplification.

One representative section from each tumor was selected for immunohistochemical staining for ER, PR, HER2neu and Ki67. Immunohistochemical testing was done by DAKO envision method according to manufacturers recommendations. The results for ER and PR were scored in a semi quantitative fashion incorporating both the intensity and the distribution of specific staining [14]. For each tissue a value designated as H-SCORE was derived by summing up the percentage of cells staining intensity multiplied by the weighted intensity of staining. An H-SCORE of less than 50 was established as negative, whereas an H-score of >50 is considered as positive for ER and PR expression.

HER2neu were scored based on the intensity and percentage of positive cells on a scale of 0 to 3+. Cases were reported 0 (negative) if no staining or membrane staining in less than 10% of invasive tumor cells was seen, 1+ (negative) if faint/barely perceptive membrane staining was detected in more than 10% of invasive tumor cells, 2+ (positive) if weak to moderate complete membrane staining in more than 10% tumor cells or <30% with strong complete membrane staining, or 3+ (positive) if strong complete membrane staining in more than 30% invasive tumor cells was seen [15].

Ki-67 immunoreactivity was recorded as continuous variables, based on the proportion of positive tumor cells (0%-100%). Besides evaluating Ki-67 as continuous variable, levels of Ki-67 were quantified as high Ki-67 (immunostaining ≥ 30%), low (immunostaining < 15%) and intermediate (between 16 to 30%) approach adopted by St Gallen International Expert Consensus [16,17].

Cases with intermediate (2+) expression of Her2neu underwent subsequent FISH testing for Her2neu gene amplification. FISH testing was performed using FDA approved Path Vysion Her2 DNA Probe kit according. Paraffin embedded tissues were cut at 5 microns and mounted on positively charged glass slides. Four slides were prepared, with one slide stained with H and E, the selection of tissue and the identification of target areas on the H and E stained slides was performed by a pathologist. Using the H and E slide as reference, target area was etched with a diamond tipped scriber on the back of the unstained slide to be assayed. Glass slides with paraffin embedded tissue sections were baked at 56C overnight. Tissue was then processed in xylene, ethanol, purified water and wash buffer according to manufacturer recommendations. Probe mixture was applied to the target area of the tissue on slide, sealed with rubber cement and then incubated in thermobrite for hybridization. After post-hybridization buffering, DAPI (counter stain) was applied. Slides were analyzed by two technologists, interpreting 60 interphase nuclei using fluorescence microscope equipped with appropriate excitation and emission filters allowing the visualization of the orange and green fluorescent signals.

Results were expressed as the ratio of Her2 signals as compared to CEP 17 signals according to ASCO/CAP guidelines. A HER2: CEP 17 ratio of less than 1.8 was considered as absence of HER2 gene amplification. A HER2: CEP 17 ratio from 1.8-2.2 was taken as equivocal and ratio of >2.2 was considered gene amplification when there were greater than 6 HER2 signals per nucleus.

## Results

Out of 1104 cases of breast cancer identified during the study period, 205 cases (18.6%) were triple negative for ER, PR and Her2neu or non-amplified on Her2neu gene amplification by FISH testing and therefore included in the study. Out of these 205 cases, 110 patients underwent primary surgery either radical or conservative while in 95 cases trucut biopsy was done followed by neoadjuvant therapy. Mean age for the patients was 48.4 years (±12.3). A significant number of cases were diagnosed at a younger age less than 50 years (60%). Very few cases were at pT1 stage (12.7%), while most of them were either pT2 or pT3. Although ductal carcinoma was the most frequent histologic type, a meaningful number of cases exhibited metaplastic and medullary like features (10.7% and 5.9% respectively) (Figure 1). Similarly geographic necrosis involving more than 40% of tumor and extensive lymphocytic infiltration was a considerable finding. Mean Ki67 index was 45.2% (±25.2) and as a reflection of tumor grade, a significantly higher proportion of cases (66.3%) were under high risk Ki67 category (>30%) as defined by St. gallen international expert consensus recommendations. Lymph node metastasis and lymphovascular invasion were seen in 48.2% and 27.3% cases respectively. Detailed clinicopathologic characteristics of the studied cases are presented in [Table 1]. Correlation of tumor size with lymph node status, Ki67 index and tumor grade are shown in [Table 2], which shows a positive significant correlation between tumor size and lymph node status. Correlation of Ki67 index with tumor size, lymph node status and tumor grade are shown in [Table 3].

**Figure 1:** **Micrographs of carcinoma with medullary features. (a-c)** Infiltrating carcinoma with circumscribed pushing borders, dense peripheral lymphoid infiltrate and syncytial growth pattern. **(d)** High Ki-67 index in tumor cells.

**Table 1:** Clinicopathologic features of triple negative breast cancers

**Variable**	**n = 205**
**Age at dignosis**	
Mean ± SD (years)	48.4 ± 12.3
**Age specific groups, N (%)**	
< 30 years	15 (7.3%)
31-40 years	47 (22.9%)
41-50 years	61 (29.8%)
51-70 years	70 (34.1%)
> 70 years	12 (5.9%)
**Tumor size**	
Mean ± SD (mm)	38.2 ± 16.2
**Size specific groups, n (%)**	
≤ 2.0 cm (pT1)	14 (12.7%)
2.0-5.0 cm (pT2)	81 (73.6%)
> 5.0 cm (pT3)	15 (13.6%)
Without surgery/trucut biopsy^$^	95
**Histological type, n (%)**	
Infiltrating ductal carcinoma (NOS)	158 (77.1%)
Infiltrating lobular carcinoma	05 (2.4%)
Metaplastic carcinoma	22 (10.7%)
Invasive papillary carcinoma	07 (3.4%)
Infiltrating carcinoma with medullary features	12 (5.9%)
Missed ductal and lobular carcinoma	01 (0.5%)
**Histologic grade, n (%)**	
Grade I (well differentiated)	
Grade II (moderately differentiated)	
Grade III (poorly differentiated)	10 (4.9%)
	65 (31.7%)
	130 (63.4%)
**Lymphovascular invasion, n (%)**	
Present	
Not present	
Cannot be assessed^$^	30 (27.3%)
	80 (72.7%)
	95
**Necrosis, n (%)**	
Geographic necrosis involving > 40% of tumor	
Necrosis involving < 40% of tumor	
Necrosis is absent	34 (30.9%)
Cannot be completely assessed^$^	72 (65.5%)
	04 (3.6%)
	95
**Lymphocytic infiltration, n (%)**	
Extensive lymphocytic infiltration	21 (19.1%)
Mild to moderate lymphocytic infiltration	89 (80.9%)
Cannot be completely assessed^$^	95
**Lymph node status, n (%)**	
Negative lymph nodes (N0)	57 (51.8%)
1-3 positive lymph nodes (N1)	24 (21.8%)
4-9 positive lymph nodes (N2)	11 (10.0%)
≥ 10 positive lymph nodes (N3)	18 (16.4%)
Lymph nodes dissection not done	95
**Extranodal extension, n (%)**	
Present	
Not present	15 (13.6%)
Lymph nodes dissection not done	95 (86.4%)
	95
**Ki-67 proliferation index**	
Mean ± SD (%)	45.2 ± 25.2
**Ki-67 proliferation index, (categories), n (%)**	
≤ 15% (low)	
16-30% (Intermediate)	
>30% (High)	32 (15.6%)
	37 (18.0%)
	136 (66.3%)
**Type of surgery n (%)**	
Modified radical mastectomy	
Breast conservation surgery	
Surgery not done/trucut biopsy	90 (43.9%)
	15 (7.3%)
	95 (46.3%)
**Laterality n (%)**	
Right	94 (45.9%)
Left	111 (54.1%)

^$^Cases are of trucut biopsies without surgery.

**Table 2:** Correlation of tumor size with lymph node status, Ki67 index and tumor grade

**Sr. no.**	**Tumor size**				
		**T1**	**T2**	**T3**	**p-value**
1.	**Lymph node status**				
	Positive	3	35	10	0.036
	Negative	12	45	5	
2.	**Ki67 index**				
	Low	4	14	8	
	Intermediate	3	18	49	0.876
	High	8	49	8	
3.	**Tumor grade**				
	GII	2	11	4	0.422
	GIII	13	70	11	

**Table 3:** Correlation of Ki67 index with tumor size, lymph node status and tumor grade

**Sr. no.**	**Ki67 index**				
		**Low**	**Intermediate**	**High**	**p-value**
1.	**Tumor size**				
	T1	4	3	8	0.876
	T2	14	18	49	
	T3	4	3	8	
2.	**Lymph node status**				
	Positive	8	14	26	0.245
	Negative	14	10	38	
3.	**Tumor grade**				
	GI	3	1	6	0.180
	GII	7	17	41	
	GIII	22	19	89	

## Discussion

Breast cancer is a heterogeneous disease encompassing numerous distinct histologic and gene profile based subtypes. Triple negative breast cancers represent one of the most aggressive phenotype with discrete risk factors and ominous prognostic significance. Our data represents the first study highlighting the clinical, histopathologic and prognostic factors of basal like breast cancers in our population.

Several studies evaluated the risk factors associated with basal like breast cancers including age, race, ethnicity, reproductive and parity history, breast feeding and obesity. Trivers KF et. al in a study involving 476 patients evaluated socio-demographic and reproductive characteristics of breast cancers. Their data revealed that hormone receptor negative breast cancers were associated with black race and young age at first birth. They also affirmed that history of recent birth and obesity as being risk factors for these cancers [18]. Phipps AL et al. suggested nulliparity as a protective factor for triple negative breast cancer, although they didn’t find a significant association with breast feeding and oral contraceptive usage [19]. Risk factors for basal like cancers were also explored in Carolina breast cancer study. They found increased parity, younger age at first term full-term pregnancy, longer duration of breastfeeding, increasing number of children breastfed, and increased duration of breastfeeding per child each associated with an overall decrease in the risk of basal like breast cancers [20]. Although we did not evaluated all these parameters in our study but we found a higher frequency of basal like cancers in reproductive age group women.

Some authors suggested that triple negative and basal like breast cancers are not entirely similar entities. Basal like cancer is a molecular defined category of breast cancer with expression of unique set of genes involving epidermal growth factor (EFGR), basal cytokeratins (CK) 5/6, proliferation gene clusters and low expression of hormone and Her2neu genes [21]. Bertucci F evaluated gene expression profile of 172 cases of triple negative breast cancers and found 72% to express basal like phenotype [22]. Gene expression profile separated out several subtypes of triple negative cancers including two basal subtypes, immunomodulatory, mesenchymal, mesenchymal stem-like, luminal androgen, claudin-low and interferon-rich subtypes [23-25]. How much these subtypes behave differently clinically is yet to be fully understood, but chemotherapy is the main stay of treatment as they are generally insensitive to targeted hormonal and herceptan therapy. Phase II clinical trials are under way to fully establish the potential role of anti-EFGR therapy in triple negative breast cancers.

Kreike B et. al in a study involving 97 triple negative cases of breast cancer evaluated clinical, histological and molecular features. They found 59% of cases were below 50 years of age and 65% of tumors were above 2 cm in maximum dimension. Although 83% of cases showed typical ductal morphology but 3 cases were metaplastic carcinomas. Concordant with our results vast majority of tumors (86%) had high grade morphology and heavy lymphocytic infiltrate was seen in only 12% of cases. They also evaluated p53 and EFGR status and positivity was seen in 50 and 27% of cases also pointing towards aggressive nature of these tumors [26].

Fulford LG et. al suggested specific morphologic features which were predictive of basal subtype. These included central scar, tumor necrosis, presence of spindle cell or squamous metaplasia, high total mitotic count (> 40 per 10 high-power fields) and high nuclear-cytoplasmic ratio [27]. We also found high grade morphology and tumor necrosis in a significantly higher number of cases.

We found a higher frequency of metaplastic histology in our study (Figures 2 and 3). Metaplastic carcinoma itself is a heterogenous group of tumors including sarcomatoid [28], squamous cell [29], adenosquamous [30], mucoepidermoid, matrix producing [31], metaplastic carcinoma with osteoclast like giant cells [32] and low grade fibromatosis like spindle cell carcinoma [33]. We encountered 10 cases of adenosquamous carcinoma, 8 of matrix producing and 4 cases of sarcomatoid carcinoma. These three categories are among the most aggressive subtypes of metaplastic carcinoma, again pointing towards the adverse morphologic characteristics of triple negative tumors. Reis-Filho JS et. al in a study involving 65 cases of metaplastic carcinoma found 91% to be of basal like phenotype irrespective of specific subtype [34]. Our results are in agreement with these findings.

**Figure 2:** **Micrographs of metaplastic carcinoma, matrix producing type. (a-b)** Tumor cells producing abundant myxoid matrix. **(c)** Microphotograph showing high Ki-67 index.

**Figure 3:** **Micrographs showing metaplastic carcinoma. (a-b)** Matrix producing type with area of necrosis.

We also found 12 cases in our study with medullary like features including high grade histology, lack of insitu component, pushing borders, syncytial growth pattern and dense lymphocytic infiltration (Figure 1). Gene expression profiling studies depicted this notion that medullary like carcinomas belong to basal subgroup inspite of being associated with a better prognosis [35].

Our study validated the strong association of triple negative cancers with tumor grade and proliferative index. Methodology of Ki67 index has not been standardized yet and different cut off points were used in different studies to designate high Ki67 index (5-30%) [36,37]. We therefore used 2 cut off points to stratify Ki67 index into 3 categories; the approach advised by St. Gallen International Expert Consensus. By categorizing Ki67 index into three categories in our study, a significantly higher proportion of triple negative cancers fell under the umbrella of high risk Ki67 index (66.3%). Spitale A. et al. in a study involving 90 basal cancers also found similar association in Ticino breast cancer registry based study with more than 75% of basal cancers having Ki67 index greater than 20% [38]. This observation is supported by high expression of proliferation gene clusters seen in gene expression profiling studies [39,40].

In our study, lymph node metastasis at the time of diagnosis was found in 48.2% of cases. Vallejos et. al in a study involving 255 basal like cancers found lymph node positivity in 54.9% of cases [41]. Blows FM et. al in a collaborative review of 1645 triple negative breast cancer subdivided them into basal and non-basal phenotypes on the basis of CK5/6 and EFGR positivity. In the basal subgroup lymph node metastasis was seen in 40% of cases while non-basal triple negative phenotype exhibited lymph node metastasis in 46% of patients [42].

A morphologic study of basal cancers in Turkish population revealed that all medullary and 55.6% of metaplastic carcinomas showed basal phenotype which is concordant with our findings. Moreover they found an increased prevalence of basal cancers in younger age group. Morphologic features associated with basal cancers in their study included high nuclear grade, increased mitotic activity, geographic necrosis, pushing border of invasion and stromal lymphocytic response. Among IHC markers, vimentin was positive in 53.2% and CK 14 in 27.7% of cases [43].

Triple negative cancers are a heterogeneous group of tumors with slightly different prognostic profiles. Therefore various markers were assessed to predict the prognosis in triple negative cancers. Markers which were found to be associated with poor prognostic profile in triple negative cancers include CARM1, TTF1 and SBEM. Coactivator-associated arginine methyltransferase 1 (CARM1) belongs to protein arginine methyltransferase family. CARM1 was found to be to be expressed in 57% of triple negative cancers and was associated with high tumor grade [44]. Thyroid transcription factor 1 (TTF1) is marker of lung and thyroid origin. Expression of TTF1 was also demonstrated in basal phenotype breast cancers. TTF1 expression was co-related with high tumor grade, lymph node metastasis and vascular invasion [45]. Similarly small breast epithelial mucin (SBEM) which has been implicated in tumor genesis and micrometastasis in breast cancer is associated with poor prognostic profile in triple negative breast cancer. SBEM expression was found to be highly co-related with higher tumor size, grade, nodal status, TNM stage and Ki67 index. Moreover multivariate analysis showed that patients with high expression of SBEM had higher risk of tumor recurrence and mortality [46]. Apart from IHC expression of various markers, role of microRNAs (miRNAs) were also evaluated in triple negative breast cancers. MiR-34b negatively co-relates with disease free survival and overall survival in triple negative cancers [47]. Laurinavicius A et. al evaluated multiple IHC markers in breast cancer. They found a high expression of p16 in triple negative breast cancers [48].

Gene expression profiling studies are not widely available in our country and cannot be performed on every case of breast cancer. Immunohistochemical studies are relatively less expensive and therefore can be performed for initial segregation of cases into specific expression profiles. Based on morphology and immunohistochemical profile, genetic studies can be performed to identify at risk families as an effective preventive measure.

Risk factors for specific morphologic subtypes of breast cancers have not been substantiated yet. Unlike smoking induced squamous metaplasia which is considered a pre-malignant change in bronchial epithelium, squamous metaplasia in ductal epithelium of breast is not considered pre-malignant. On the other hand, as most of the metaplastic carcinomas have been showed to harbor basal phenotype, underlying BRCA mutations and familial predisposition may play a role.

We analyzed 1104 breast cancer patients, out of which 205 cases exhibited triple negative phenotype with a frequency of 18.6%. Compared to international data, only Chinese, African Americans and Peruvians had a greater frequency of triple negative cancers than ours with a figure of 21.5%, 21.5% and 21.3% respectively [11,49]. The frequency of triple negative cancers in Caucasians, Australians and UK population was found to be low with a frequency of 12.5%, 14% and 13% respectively [50,51].

Another significance of basal like breast cancers lies with its association with BRCA 1 mutations. It was shown that, more than 80% breast cancers occurring in women with BRCA 1 mutation have a basal like profile. Although most basal cancers are sporadic, they are also associated with an abnormal BRCA 1 pathway [52-54]. Although young age breast cancers are quite prevalent in our population, however genetic testing including BRCA mutations were not widely done in our population. Therefore we suggest that risk factors associated with triple negative breast cancers especially those occurring in a younger age group with metaplastic and medullary histologies should be sought including underlying BRCA 1 mutations. In addition evaluation of EFGR mutations and potential role of EFGR therapy in basal like cancers should also be addressed.

## Conclusion

Triple negative breast cancers typify high grade breast cancers with a higher frequency of atypical medullary and metaplastic histologies. Their prevailing occurrence at a younger age raises question of under lying BRCA mutations in our population. Therefore, we suggest that risk factors including BRCA 1 mutations should be uncovered in reproductive age group breast cancers especially those disclosing basal like phenotype.

## Competing interests

The authors declare that they have no competing interests.

## Authors’ contributions

AAH: main author of manuscript, have made substantial contributions to conception, design and acquisition of data. MME: main author of manuscript, have made substantial contributions to conception and design, or acquisition of data, or analysis and interpretation of data. HN: revising it critically for important intellectual content. NF: revising it critically for important intellectual content. AK: have given final approval of the version to be published. MK: have been involved in drafting the manuscript or revising it critically for important intellectual content. All authors read and approved the final manuscript.
